RETRACTED

# A Study of the Political Culture of the Ming and Qing Agribusiness Societies under the Imperial Environment

**DOI:** 10.1155/2022/5367271

**Published:** 2022-06-28

**Authors:** Guiling Yuan

**Affiliations:** Department of Literature and Law, Science and Technology College, Gannan Normal University, Ganzhou, Jiangxi 341000, China

## Abstract

In the Ming and Qing dynasties, while the social life, economic structure, and even cultural atmosphere underwent profound changes, the dominant aspect of political culture was still deduced along the traditional track of the imperial system. The prominent characteristics of China's social form in the Ming and Qing dynasties are the development of the commercial economy and the enhancement of social freedom; the developed trend of common people's culture; and the sustainable development of the centralized monarch-bureaucratic-aristocratic system, which constitute a self-consistent pattern. This paper on the political culture of political spirit, political value, political thought, the four dimensions, the specific period, specific social community, public power setting and operation, and the perspective of the Ming and Qing social form of political culture, this study helps people to the imperial environment of Ming and Qing rural political culture and understanding and exploration.

## 1. Introduction

The study of political culture should include the investigation of the setting and operation of public power in a specific period and a specific social community from the four dimensions of political spirit, political value, political thought, and political ecology [1]. Before the Ming and Qing dynasties, the main political structure of the central government is shown in Figure 1.

However, in the Ming and Qing dynasties, while social life, economic structure, and even cultural atmosphere underwent profound changes, the dominant aspect of political culture was still deduced along the traditional track of the imperial system. The centralized institutions of the Ming and Qing dynasties are shown in Figure 2. The prominent characteristics of China's social form in the Ming and Qing dynasties are the development of the commercial economy and the enhancement of social freedom, the developed trend of common people's culture, and the sustainable development of the centralized monarch-bureaucratic-aristocratic system, which constitute a self-consistent pattern. This self-consistent pattern shows the potential of the imperial rural business society to continue to extend under the prosperity of the commodity economy [2]. The conflict between China and the west in the mid-19th century was not the meeting of two societies at different stages of the same historical process, but the intersection of two civilization systems in different historical processes in the spatial and temporal pattern of the Asian continent [3].

RETRACTED

In the rural and commercial societies of the Ming and Qing dynasties, the political culture in the imperial environment is mainly reflected in the political spirit. Political thought is the rational understanding of political phenomenon on the basis of political experience and political perceptual understanding, and it is the abstract and logical explanation of the internal causal relationship of political phenomenon and its development law. Political thought is a systematic, complete, and rigorous political thinking achievement and ideology, usually composed of political thought, political belief, and political theory.

Institutions embody the rigid statutes of the dominant groups in society to keep society in a certain state, among which the most public power and political attributes are the basic institutions of the state [4]. Human history has shown a variety of state institutions, including various monarchies, feudal systems, constitutional monarchies, republics, presidential systems, cabinet systems, parliamentary systems, and so on, as well as a variety of mixed and variant forms. The construction of all these basic institutions of the state reflects the expectations, concepts, and demands of the dominant people in a given social community regarding the establishment and operation of public power [5]. The spirit of politics, as a fundamental area of political culture research, is to look behind the rigid structure of the basic institutions of the state to understand their expectations, ideas, and demands to achieve an understanding of the inner rationale and the real and potential tendencies of the political system of concern, as well as an understanding of the universal meaning of a specific political system.

In the Ming and Qing dynasties, China was not a legal or constitutional state, so the basic institutions of the state at that time were not entirely defined by the texts of laws and regulations, but rather by a combination of texts of regulations and the derivation of governance. Specific changes occurred frequently, but the fundamental regulation was consistent [6]. The axis of the public power structure was the emperor-bureaucrat-county system. This system, gobbled up in the earring states, was customized in the Qin and Han dynasties, and in the Yuan dynasty, there were provinces as a large regional hierarchy between the central government and local administration, which continued unchanged until the Ming and Qing dynasties. In contrast to the colorful changes in the economic and cultural fields, the aforementioned basic structure of the Ming and Qing dynasties has a long history and shows no definite signs of change in a practical sense. In the sense of ideology, the clearest movement was the criticism of the privatization of the monarchy expressed by Huang Zongxi in the early Qing dynasty in his Ming Yi Zuoren. Huang's proposal, however, could only reach the level of co-rule of monarchs and ministers and did not consider or propose the abolition of the monarchy, nor could it propose a constitutional system of monarchy [7]. Moreover, Huang's book became taboo before it was published and did not see the light of day until the late Qing dynasty, and did not have a substantial impact on the trend of the political spirit of the Chinese state in the Qing dynasty. With regard to the bureaucratic-provincial-county system, the Ming and Qing dynasties practiced a centralized system of states and regions under the provincial authority in the core areas: the thirteen prefectural administrations in the Ming dynasty and the eighteen provinces in the Qing dynasty, without change [8]. This inheritance of the basic system from previous eras indicates a tendency for the political system to remain “unchanged,” which in turn indicates that the dominant public power in the Ming and Qing dynasties did not take into account the need for the political system to change with the times, as shown in Table 1.

RETRACTED

The system of state power in the Ming and Qing dynasties was not fixed, but it was not in the category of fundamental institutions.

As for the late Qing dynasty, there were many institutional changes in a substantive sense, but already after the external challenges and comprehensive crisis. Therefore, to read the spiritual qualities of the Chinese public power system in the Ming and Qing dynasties, imperial power politics, bureaucratic scholar politics, and aristocratic politics are three keywords [9].

## 2. Political Values

The so-called political values refer to social members' conceptions about the meaning and contingency of political systems, political life, and political phenomena. The social and political value of rural agriculture and commerce in Ming and Qing dynasties mainly includes the three aspects shown in Figure 3. Such conceptions determine at a deep level the attitudes and psychology of social members toward the established public power settings and their operational states. Such attitudes and psychology may be expressed in verbal and textual ways, or in nonverbal and textual ways during various opportunities and occasions of life practice [10]; for example, in all societies, the members of the society expect the government to organize to keep the society free from external forces, the government that cannot do this will surely perish; the members of all political societies expect the government to bring order, the government that cannot bring order will be replaced; most members of all political societies expect their governments to maintain social justice, although in fact it is difficult for society to be completely just, it is difficult to maintain a society without justice. Many political conflicts throughout history have been not only conflicts of interest but also conflicts of values. From the perspective of political values and the basic attitudes of members of society toward political life, the following issues in particular need to be considered in the Ming and Qing dynasties [11].

RETRACTED

### 2.1. National Consciousness

National consciousness is one of the common psychological qualities and one of the national characteristics. It refers to the psychological state embodied in the characteristics of national culture in the process of formation and development. What members of society think the state is, how the state is related to their own existence, and what is the basis and shape of their identification with the state are all elements of political values. The state consciousness of the mainstream people in most of the Ming and Qing dynasties was the consciousness of the subjects [12].

The core of this consciousness was obedience to the imperial court, which was the “Emperor of Heaven.” If the court's governance led to the people's unhappiness, the people might take the risk of rebellion; if the court completely lost its virtue and power, the walls would fall down and the people would push, and they would establish or change to a new dynasty; in case of foreign invasion, if the court could function normally, they would participate in the court to defend the country from the enemy. In the Ming dynasty, all of the aforementioned situations occurred, and the people's attitude toward the state did not differ significantly from that of previous generations. In the late Ming and early Qing dynasties, the Qing army entered and moved southward, and while achieving the reunification and cultural integration of the national community, it introduced forced changes in culture and customs, which not only met with resistance from the remnants of the Ming dynasty but also provoked direct resistance with the active participation of a large number of southerners [13]. After the suppression of the large-scale armed resistance movement against the Qing dynasty, the activities of anti-Qing secret societies continued unabated until the late Qing revolution. This situation reflects the more complex entanglement between national identity and national cultural identity and the conflicting interests of groups. During this period, the enlightenment of the national view of the state may have occurred with reference to the idea of defining the state by cultural identity expressed by Huang Zongxi, Gu Yanwu, and Wang Fuzhi in the early Qing dynasty, but comparing the early Qing dynasty with the early Yuan dynasty, it is not certain whether a new qualitative situation of national consciousness really occurred at the level of popular and popular psychology in the early Qing dynasty. At the same time, the mainstream of the Qing people, and even the gentry and business class, actually gradually accepted the legitimacy of the Qing dynasty. Otherwise, it would be impossible to account for the nearly 270 years of the Qing dynasty's national movement [14]. This process, because the change of regime in the Ming and Qing dynasties was accompanied by national conquest, made the process of general acceptance of the early Qing regime slower than the same process in the early Ming dynasty. The gradual social acceptance of the Qing dynasty was due to the prevailing subject consciousness of the people under its rule as the primary factor. A population dominated by the subject consciousness was politically passive, with survival as its basic demand, and lacked the capacity for collective behavior, tending not to confront the real rulers when possible [15]. The measures taken by the Qing government to adapt to the culture of the middle Kingdom and to collect the hearts and minds of the people were the second factor at play. The administrative effectiveness of the early Qing government in contrast to the late Ming government and the effectiveness of its governance was the third factor of action that gradually emerged. The rise of a new national consciousness after 1840 was a huge difference from any previous era, but it could not occur without the challenge of western colonialism and the impact of western ideas, so it does not prove that it occurred within the logic of the Ming-Qing imperial peasant-merchant society itself. To sum up, if we want to inquire into the changes in state consciousness during the Ming and Qing dynasties, we should focus on the time of the Qing rather than the Ming. Although the Qing and Ming dynasties are referred to as “empires” in many researchers' vocabulary, especially in western scholarly works, the nature of the Ming dynasty is lighter and the Qing dynasty is clearer, the Ming dynasty was essentially a local state, while the Qing dynasty united the vast majority of the territory and people of the traditional Chinese civilization. This change must have had some impact on the state consciousness of the nobility and the scholarly officials, and probably had a similar impact on the state consciousness of the people. Whether such effects were closer to a “modern” nation, state consciousness in any sense of the word than to the state consciousness of previous generations requires further analysis [16].

RETRACTED

### 2.2. The Concept of Political Legitimacy

Political legitimacy refers to the legitimacy or legitimacy of the government based on the principle recognized by the public. To put it simply, to what extent the government is regarded as reasonable and moral by the citizens. Politics is a system of coercive power that operates to gain legitimacy, and coercive power itself can only constitute an integral part of the state management function on the basis of gaining social legitimacy identity, otherwise, it is only order subversive power. The political power, the supreme ruler, and the major decrees are legitimate under what circumstances, and the political behavior of which people is legitimate, which constitute the bottom line of the operation of the public order of the political system. However, the term “legitimacy” here is a discourse of ideas and psychological tendencies, mainly referring to the orthodoxy, legitimacy, and rationality of political rule, rather than whether it conforms to the attributes stipulated in legal texts.

The legitimacy of state power in the Ming dynasty was repeatedly affirmed by the Ming rulers and ministers, the core of which was first, to accept the fate of heaven; second, to sweep away the Hu customs; and third, to return the four seas to the heart. This is repeatedly seen in the various imperial edicts and documents of the early Ming dynasty. To simplify it, it means the will of heaven, the hearts of the people, and cultural inheritance. The first two, certainly entirely traditional in nature, with the restoration of Chinese clothing as the basis for the legitimacy of the Ming dynasty's statehood, had the novelty of the times. In China, before the Yuan Dynasty, although there was a nomadic regime established by nomads, there was no unified nomadic regime. The rule of the Yuan Dynasty may fundamentally change the direction of Chinese cultural evolution. Therefore, the founding of the Ming dynasty had the significance of “restoration” in terms of the cultural circle of the central plains [17]. This gave the early Ming dynasty an additional layer of legitimacy. However, as a result, the Ming dynasty also became a localized state, with less control over the peripheral regions outside the traditional Han areas. Such affirmations by the Ming government had certain repercussions in the popular psyche. Traces of this can be seen in the gradually increasing literature of the common people from the mid-Ming period onward. The social recognition of the legitimacy of Qing rule encountered a much greater obstacle than that of the Ming.

RETRACTED

In order to remove this obstacle, the rulers of the early Qing dynasty, in addition to declaring that they would be the first to accept the fate of heaven and that the four seas would return to their hearts, announced policies such as crushing the “rogue thieves” for the Ming dynasty, consecrating the Ming tombs, and recruiting Confucian scholars and thinkers to serve in the government, inherited the basic institutions and laws of the Ming dynasty, accepted the upper-class culture of the central Plains, and also, by launching a written prison, suppressed the forces that refused to agree with the legitimacy of the Qing dynasty. They also suppressed the forces that refused to agree with the legitimacy of the Qing dynasty by initiating written jails, etc., and very seriously reevaluated the relationship between rulers and subjects and between China and yi [18]. In the long-term process of moving from general resistance to mainstream identification with Qing rule, force and wai-yi tactics were the main factors initially; gradual stabilization of people's livelihoods and gradual cultural integration were the main factors later. This suggests that the establishment of regime legitimacy in the early Qing dynasty was, in fact, not fundamentally different from the logic of earlier eras. However, it is still important to see that the revolutions that took place during the late Qing dynasty, including the failed Taiping heavenly kingdom and the partially successful Xinhai revolution, all raised the banner of hair storage or anti-Manchu, and the psychology of the Qing dynasty as a conquering ruler has never completely disappeared, meaning that the legitimacy achieved by the Qing dynasty has been limited. The majority of the public thought that the government's rule (including the threat of force) was improper, so the concept of political legitimacy was restricted in the Qing dynasty.

Closely related to political legitimacy is the notion of political rationality, both have a significant influence on political culture, that is, the sense about whether political initiatives are in line with basic political value concepts. For example, the early Ming and early Qing dynasties both had written prisons, which were never endorsed as reasonable in the public psyche or even in the official historical accounts afterwards. The eunuchs' control of the imperial government also never gained public approval. The late Ming emperors sent mine supervisors and tax ambassadors and the court to suppress the Donglin party, which had aroused public anger. Qing officials and honest officials, both in the Ming and Qing dynasties, became a group of people expected and praised by the public. However, the political concepts that can show these phenomena can still be found in the political and cultural traditions of the previous era, and it is difficult to determine, which have been new political and cultural factors.

RETRACTED

### 2.3. The Sense of Political Participation

Political participation is a great progress in China's political democracy and also an important embodiment of the concept of “people-oriented” in the field of political life. This is an important concept in Almond and others' analysis of political culture in modern democracies. Ming China was not a democracy, and thus members of society were certainly less enthusiastic about participating directly in politics than the societies Almond examined. Even so, any functioning political system involves the question of whether and to what extent and in what manner members of society participate. In times of nonrevolution, turmoil, war, and frenzy, the enthusiasm of people's political participation are proportional to the public nature of the operation of political power. If the degree of Chinese political participation in the Ming and Qing dynasties was higher than in previous eras, it may mean that the openness and public nature of this social system increased, and if it did, it tended to be more modern in nature. The main group of people who directly participated in politics in the Ming dynasty were intellectuals, whose preparation stage was to study and join the imperial examinations; and after the imperial examinations, they joined the government and thus entered the national political trend. Another way of political participation for this group of people is to lecture in the field. There were lectures in the middle and late Ming dynasty, some of which were lectures by intellectuals with the status of a scholar, and some were lectures by intellectuals in cloth without the status of a scholar. At that time, the so-called lectures, there is no knowledge of science as it is called today, are sincere in ruling the country and the world. Whenever it comes to current affairs, it has the nature of political participation [19].

The sense of political participation among members of society in the early Qing dynasty was not more positive but more negative compared to that of the Ming dynasty. This is certainly related to the ethnic conflicts that developed during the Ming-Qing transition, as well as to the longer and harsher writing prison that lasted in the early Qing dynasty. Under the influence of the literary prison, the average number of Jinshi admitted in the Ming and Qing dynasties changed greatly, as shown in Figure 4. At the level of the scholarly class, the Qing dynasty did not have the private lectures that used to be prevalent in the Ming dynasty, where commenting on current affairs was an important element, nor did it have the phenomenon of confrontation between rulers and ministers on a very large-scale. The party movement of the scholarly class ceased, and was replaced by the secret society of the civil society, which was more prevalent than in the Ming dynasty. The former was open and thus reflected political participation based on recognition of the existing system; the latter was secret and thus reflected political hostility based on nonrecognition of the existing system. It was only after the mid-19th century that the situation changed radically.

RETRACTED

## 3. Political Ideology

Political thought is related to political values, ideological, and political education value is a utility relationship between the needs of subjects and the attribute of the object. Socialist core values, as the guidance and foundation of ideological and political education value, play an irreplaceable role in promoting the realization of ideological and political education value. As human essence, ideological and political education practices the socialist core values, and the two are dialectically unified in the process of the realization of ideological and political education value. But political thought is more often embodied in explicit claims expressed through language and texts than in political ideas embodied in emotions, attitudes, and behaviors that are either clear or vague. Generally speaking, to grasp the basic face of political thought in an era, one needs to examine the discourses of thinkers in that era. Therefore, the history of political thought always carries the implication of elite history. The history of ideas is the core part of cultural history, and political thought is also the core part of political culture, and its significance in the study of political culture is self-explanatory. The two most accomplished researchers in the study of traditional Chinese political culture, Yu Yingshi and Liu Zehwa, as mentioned earlier, have paid special attention to the elements and clues that can constitute “ideas” in their research, as shown in Table 2.

In the political thought of the Ming and Qing dynasties, the ideas that gained practical status were, first of all, the political outlook of authoritarian imperialism, which was prominently reflected in the statements of Zhu Yuanzhang in the Ming dynasty and the Kangxi, Yongzheng, and Qianlong emperors in the Qing dynasty, including the edicts and the chapter and verdicts [20]. The second is the people-oriented political doctrine of later Confucianism. The aforementioned monarchs and Confucian scholars and thinkers in politics were in general agreement on the basic institutions of monarchy, bureaucracy, centralization, and limited aristocracy, but diverged on the issue of the limits and constraints of imperial power. The scholars and thinkers of the Ming dynasty had been trying to keep imperial power regulated to a certain extent, seeking to expand the scholars' voice in the political operation of the state; the Qing dynasty's scholars and thinkers had been trying to expand their power to a certain extent. In the Qing dynasty, the scholars abandoned this effort and converted to the absolute authority of imperial power. According to such basic clues, Zhu Yuanzhang was the first representative of imperialist thought in the Ming dynasty, and the subsequent emperors were all on the path of their practice, but rarely had new ideological expressions of the nature of invention and elaboration. The three emperors of the Qing dynasty, Kangxi, Yongzheng, and Qianlong, are the representatives of Qing style imperialism. They did put forward some political ideas with new meaning based on their admiration of Zhu Yuan zhang's political thought and political action.

RETRACTED

In order to more clearly view the role and development of political thought in the Ming and Qing dynasties, it is necessary to introduce the study of Confucian political thought in the Song and Ming dynasties.

It is the fact that Confucian political thought in the Song and Ming dynasties was people-oriented in terms of value goals, i.e., it took the state of people's livelihood as the measure of political legitimacy and rationality rather than the interests and wishes of the monarch; in terms of institutional thought, it was based on the monarchical-bureaucratic political base, i.e., it fully recognized the monarchy and bureaucracy, as well as a limited aristocracy. On this basis, the political thinkers of the scholars in the early and mid-Ming dynasty did not put forward any particularly innovative ideas based on the political thought of the Song dynasty but only made some technical discussions from the perspective of how to effectively practice the Confucian political philosophy. In the late Ming and early Qing dynasties, Gu Yanwu, Huang Zongxi, and Wang Fuzhi represented the culmination of political system introspection and political philosophy criticism. Of course, their thoughts are still Confucianists in the basic direction, but in response to the lessons of the fall of the Ming Dynasty, they all more sharply advocated the people-oriented political principle, and more fiercely attacked the absolute power of the monarch, and put forward the idea of restricting the monarch's power. However, they could not and did not go beyond the basic pattern of monarchy and bureaucracy. After the Qing dynasty, the independent consciousness of the scholars quickly encountered the impact of the trend of absolute monarchical power, the late Ming and early Qing dynasty political criticism and political introspection stifled, independent political ideas such as flowers and water, so the political thought of the scholars can only be attached to the emperor's political rhetoric. Such a situation extended until the middle of the 19th century. As a result, the political thought of the Ming and Qing dynasties had hardly made any new progress. As for the basic ideas of so-called “modern” politics, such as “democracy,” “freedom,” and “rights,” and as for the so-called “modern” political ideas, such as “democracy,” “freedom,” “rights,” and “rule of law,” they could not be developed in the original political concept in the same direction, and could not become clear ideological tools without a more profound transformation of the general shape of society or interaction with the outside world.

RETRACTED

## 4. Political Ecology

The term ‘political ecology' is more specific. I mainly involve only two relevant levels here: one is the orientation of the dynasty and the other is the nature of the imperial power. It is the decline of imperial power, the power of scholar-officials, and the retreat of the sense of responsibility as the basic clue.

Political ecology refers to the general atmosphere, states, and deduction tendencies of a specific political community unfolding in its operation. The so called political history is in fact the course of deduction constituted by the succession of particular states, the state of each particular moment being the basis of the state of the next moment, and all political states being the consequences of the deduction of their previous states. The total state of a functioning political body contains the greater possibility of some political phenomena occurring in the near future, and the lesser possibility or impossibility of some other political phenomena occurring. Political ecology is naturally closely related to political institutions, ideas, and values, and at the same time is political from the perspective of the integrated dynamics of political operation, and thus does not cover institutions, ideas, and values, and deserves special scrutiny.

RETRACTED

Looking at the history of the Ming and Qing dynasties from the perspective of political ecology, we can not only see the continuity of the two generations but also the fracture of the two generations, as shown in Table 3. The most prominent the continuity is obviously the basic dynamics of the political enhancement of imperial dominance. The abolition of the prime minister in the 13th year of Hongwu, who had already existed during the pre-Qin period and had been the main person responsible for the daily administration of the central government since the Qin and Han dynasties, was a huge change. Huang Zongxi's claim that “the absence of good governance in the Ming dynasty began with the dismissal of the prime minister by the high emperor” was not a false statement, but it transformed the system, in which the emperor mainly handled major decisions and left the day-to-day administration to the bureaucratic system into one, in which the emperor was the “sole arbiter” of both decisions and administration, thus instrumentalizing the bureaucracy of the scholar and the emperor's personal will to a greater extent. If we combine this change with the action of dividing the kings in the early Ming Dynasty, which led to a short upsurge of aristocratic politics, then the strengthening of imperial power based on families in the early Ming Dynasty paved the way for the political ecology of the whole Ming Dynasty. However, the Ming dynasty, imperial power was not continuously strengthened, and the cabinet system actually provided a certain degree of institutional opportunities for the political expansion of the scholar, thus creating a complex entanglement and resistance between the two tendencies of imperial power absolute and scholarly discourse in the political history of the Ming dynasty. The admonition of Zhengde's southern tour, the great Rites, the protest against Zhang Juzheng's seizure of love, the east forest's discussion of politics, and the antimining taxation supervision, all have such implications. When investigating the political ecology of the Ming Dynasty, Mr. Yu Yingshi tried to investigate the relationship between imperial power and literature, but he only grasped the comparison of Zhu Xi's and Wang Yangming's thoughts, and did not pay attention to the above practice. He believed that scholars in the Ming Dynasty had retreated from pursuing “inner sage” and “outer king” to pursuing “inner sage,” which was an oversight. In the early Qing dynasty, imperial power was substantially strengthened for the second time.

Compared with the Ming dynasty, the important “fracture” during this period is mainly the Qing dynasty in response to the extension of the multi-ethnic state system, bringing “the first Chong Manchurian” ethnic rule color and more active management of frontier areas. This situation, from the point of view of laying down the map of modern China and promoting the integration of various ethnic groups in the Chinese civilization sphere, is of great historical progress, but from the point of view of political and cultural improvement, it is retrograde. The political science involvement is too complex to discuss briefly. Moreover, the resurgence of aristocratic politics in the early Ming dynasty soon came to an end, while the resurgence of aristocratic politics in the early Qing dynasty continued for a long time and still constituted a realistic system until the late Qing dynasty. This in turn reflects the differences between the politics of the Ming and Qing dynasties.

RETRACTED

Based on the above general observation and looking at the specific level, the most prominent situation at the temple politics level is that the active politics of the scholars in the Ming dynasty was lost until the Qing dynasty. There was active political criticism, party movements, and even confrontation between rulers and ministers in the temple. This was the last period of active scholarly politics in imperial China. Then, after the Qing dynasty, there was no longer a group of scholars to resist the imperial order, and the instrumental significance of the scholars in the temple politics increased. Thus, the whole temple politics level, forming a period of great prosperity of imperial politics. This great prosperity of imperial politics was in fact a facet of the Kang, Yong, and Qian dynasties. The politics of the scholars did not directly imply good politics, but the biggest drawback of the politics of the imperial era that could not be eradicated was the absolutization of the emperor's power. The tendency of the emperor's power to be absolute constituted a daily check. Technically, this would have increased the cost of politics, but without such a check, the social costs of absolute imperial power would have been even more profound. However, if modern researchers attach the Ming scholars' demand for restraint of imperial power to the political demand for “democracy,” it is difficult to get the point. The political aspirations of the Ming and Qing scholars, even in their most radical manifestations, were not democratic, but rather monarchical-bureaucratic politics based on people's livelihoods. The concept of the foundation of democracy, as shown in modern Western history, has not been sorted out into an ideological discourse in traditional Chinese political culture, and thus cannot be brought together into a logic and theory of thought. The modern democratic system is not a hazy feeling or tendency, but a systematic institutional pattern and profound political and cultural state, which must be developed with the help of rigorous and grand theories. The scholars of the Ming and Qing dynasties did not have this ability, and other people did not have this ability. Moreover, throughout the Ming and Qing dynasties, it is impossible to see which group of people has the possible tendency to continuously enhance this ability. V. social formation of Ming and Qing dynasties in the perspective of political culture.

RETRACTED

First, the Chinese imperial system had a high degree of tolerance for the development of the commodity economy. The rapid development of the commodity economy during the Ming and Qing dynasties prompted the imperial state system to make a number of policy adjustments, and such policy adjustments led to structural changes, such as the shift from a fiscal system based on physical goods to one based on money. Regardless of the complexity of the evolutionary process, these adjustments and changes boiled down to a basic rapprochement between the imperial system and the new economic situation of the growth of the commodity-money economy, thus presenting the peak of simultaneous prosperity of the commodity-money economy and the imperial system. This suggests that the Chinese imperial system was not in direct opposition to the general development of the commodity-money economy, but had more room for accommodation. The hypereconomic coercion of the imperial system constituted some limitations on the highly developed commodity economy, but this was only one side of the function of the imperial system; the other side was that the imperial system was also able to provide some favorable conditions for the development of the commodity economy, at least compared to the hierarchical and feudal political system. The imperial system's social control and ability to coordinate and act in a unified manner in response to external challenges exceeded that of the hierarchically divided system, requiring a large geographic deployment of manpower and materials, and thus some degree of compliance with the market economy. The basic features of the imperial era, such as a unified currency, transportation facilities, social security covering a large geographical area, and the existence of metropolises, also constituted the conditions for a developed commodity economy and market. Thus, the Chinese imperial system was not susceptible to a process of disintegration in the context of the general development of the commodity economy, nor was the natural economy of self-sufficiency a fundamental feature of the system.

RETRACTED

Secondly, the evolution of political culture in the Ming and Qing dynasties has always been entangled between change and unchanged, and there is no new political culture trend of breaking through the imperial ideology. Some innovative political ideas and concepts stimulated by the development of commodity economy are dissolved in the framework of the imperialist ideology, or shaded by the imperialist ideology. The reason for this may be related to the development that the commodity economy has not reached a sufficient level.  Figure 5 shows the economic development trend of ancient China, but more certainly, because the political culture is rooted in a deeper level of tradition. This era even the most radical thinkers, also must adopt the concept of Confucianism to think about real problems, guided by the connotation of Confucianism, and the most valuable Confucian political orientation, and imperial system has formed in the long-term historical evolution of many ways, so not enough to provide system update systematic ideas.

## 5. Conclusion

From the perspective of politics and culture, this paper intends to analyze the spirit and psychological characteristics of public power operation in China in the Ming and Qing dynasties, in order to deepen the understanding of the comprehensive characteristics and evolution tendency of the Ming and Qing dynasties. And from the perspective of political culture, this paper presents this pattern and makes a preliminary discussion, so as to discuss the characteristics of social form and trend of the Ming and Qing dynasties in the future.

## Figures and Tables

**Figure 1:** Centralized structure before the Ming and Qing dynasties.

**Figure 2:** Centralized structure of the Ming and Qing dynasties (the emperor directly commanded the six departments).

**Figure 3:** Social and political value of rural business in the Ming and Qing dynasties.

**Figure 4:** Changes of the average annual number of Jinshi in the Ming and Qing dynasties.

**Figure 5:** Economic development trend chart of ancient China.

**Table 1:** Changes in the state power system in the Ming and Qing dynasties.


1	The abolition of the prime ministerial system in the early Ming dynasty, a movement leading to the strengthening of imperial power

2	The cabinet system formed in the Ming dynasty, which is the abolition of the prime ministerial system around the functioning of imperial power gradually occurred after the compensation system, the end of the Ming dynasty has failed to exist in name only until the Qing dynasty

3	The establishment of the Qing dynasty's pre-fan court and the implementation of land conversion in the southwest were implemented in response to the expansion of the Qing dynasty's direct control over geographic space and were adaptations of the existing centralized power and provincial system in the interior to the outer edge of regional management

4	The office of military affairs became the main operating department of central power, a reflection of the further strengthening of imperial autocracy in the Qing dynasty

5	A series of systems related to Manchu privilege, such as the eight banners, the full official shortage, etc., is essentially a return to the system of aristocratic privilege

RETRACTED

**Table 2:** Some political ideas with new ideas in Ming dynasty.


1	The rhetoric about the Chinese and the Japanese as one family, as represented in the Danyi Juezhu. This idea was adapted to the expanded geographic, ethnic, and demographic scale of the multi-ethnic state, arguing for the legitimacy of Qing rule, and expressing the idea of the rationality of a multi-ethnic state

2	The unprecedented esteem for the absolute rationality of imperial rule, which is intertwined with the practice of Manchurian ministers calling themselves minions to the emperor. This shows a tendency to see from the perspective of political thought from the strengthening of monarchical dictatorship to absolute strengthening.

**Table 3:** Characteristics of the secondary reinforcement of imperial power.


1	Through the prison of words, crackdown on cronies, etc., to break the sense of autonomy of the scholars and drive away the bureaucratic tools and even slavery mentality

2	Resurrect the aristocratic politics more substantially, with the participation of the Manchu aristocracy in politics as a complement to the imperial power, offsetting the institutional status of the Shih Taishu bureaucracy

3	The emperor was diligent and the use of secret folding, court mail, and other management methods, directly weakened the voice of the scholar, to achieve the effective control of the imperial power over the entire decision-making and administrative process

## Data Availability

The labeled dataset used to support the findings of this study is available from the corresponding author upon request.
